# Immersive VR Network Management Analysis considering Automatic Topology Discovery Algorithms

**DOI:** 10.1155/2022/3625502

**Published:** 2022-09-02

**Authors:** Jing He

**Affiliations:** College of Artificial Intelligence and Big Data, Chongqing Industry Polytechnic College, Chongqing, China

## Abstract

In order to make up for the deficiency of a two-dimensional user interface, enhance the visualization of network information, and comprehensively and effectively improve the efficiency of network management, this paper attempts to use virtual reality technology to design the network management system and uses the research results of related fields for reference to carry out the specific practice, providing a new idea for the design and development of the network management system. The automatic topology discovery algorithm is introduced into the network management analysis, and the immersive network management is modularized by using the method of dividing subnets. Finally, the test results show that through the functional design of the system and the hierarchical description of the structural model, the practical method is given. Finally, the operation process of the simulation system is analyzed in detail. The proposed method can effectively reduce the network load and reduce the network bandwidth and greatly improve the slow convergence of the penetration VR network topology.

## 1. Introduction

Due to the unsustainable network hardware conditions, the automatic topology discovery algorithm network will cause more difficult problems. In the automatic topology discovery algorithm, the current primary task is the smooth propagation of network virtualization mapping. Through the establishment of nodes in the network to form multiple network transmission channels, the storage rate of network multimedia transmission data is higher, and the reliability of transmission is ensured by the form of storing the transmitted data. With the continuous development of science and technology, tremendous changes have taken place in the field of computer internet. The scale of multimedia internet has become more and more powerful, and its structure has become more complex. As the structure of the multimedia internet has become more complex, this change has made the routine control, daily management and maintenance, and data analysis of the internet more difficult. Immersive VR network management analysis provides a means for searching the network characteristics of the internet in the actual environment. Immersive VR network management analysis is also a process of effective data collection, data decoding, and data analysis for network devices. We mainly collect indicator data from the network and feed it back to the monitoring personnel. Immersive VR network detection and real-time risk warning are of great significance to the distribution of multimedia network-related resources, traffic plan service levels, and security warnings [1, 2].

Through the above analysis, this paper proposes an immersive VR network management analysis based on the automatic topology discovery algorithm. Due to certain restrictions on network resources, path segmentation cannot be performed. The automatic topology discovery algorithm is used for immersive VR network demand analysis. Constructing a binary combinatorial optimization model based on the underlying network node and link-related constraint relations can effectively realize the basic four-level mapping of the underlying network resources, and at the same time can reduce the underlying network overhead and time spent, thereby improving immersive VR network virtualization mapping success rate, revenue, and resource utilization.

## 2. Related Algorithms and Analysis Processes

### 2.1. Automatic Topology Discovery Algorithm

*Pheromone concentration*. If the set*S*is used to represent all the nodes in the immersive VR network, and the set*N*_*a*_represents the adjacent nodes of node*a*, when node*b*is in the adjacent link corresponding to node a, then the pheromone concentration*T*_*ab*_(*t*) represents the time*t*. At this time, node *a*(*a* ∈ *S*) can choose to use node *b*(*b* ∈ *N*_*a*_) to realize the jump to the next node. According to the pheromone concentration value of the link lab formed by node a and node *b*, this value the condition that needs to be met is greater than or equal to zero, that is, *T*_*ab*_(*t*) ≥ 0.

For the information data target *c*_*a*_ and the movable object *c*_*b*_ in its adjacent area, the Euclidean distance calculation method can be used to calculate the similarity of its average data. Euclidean distance can be used to represent the geometric distance between two adjacent points in a multidimensional space [3, 4]. The calculation formula is expressed as follows:

(1) $$\begin{array}{c} d\left(c_{a},c_{b}\right)=\sqrt{\sum_{k=1}^{n}{\left(c_{ak}-c_{bk}\right)}^{2}}. \end{array}$$

In the formula, *n* represents the number of attributes, and then, the Euclidean distance can be used to more vividly see the degree of similarity between the obtained data information. If the similarity value is smaller, the data objects are more similar.

Figure 1 shows the simplified structure of the pheromone diffusion model. It is supposed that point *C* indicates that the maximum pheromone concentration value is represented by *P*_max_, and the parameter is represented by a fixed acute angle. It is assumed that *CG* is used to represent the cone height, and the acquired pheromone concentration diffusion range is *CG* · tan*α*. If *β* is used to represent the distance between point *F* and point *C*, then we use formula (2) to calculate the following pheromone concentration value *P*_*f*_ at point *F*:

(2) $$\begin{array}{c} P_{f}=\frac{CG\cdot \tan\alpha -\beta }{CG\cdot \tan\alpha }\cdot P_{\max}. \end{array}$$

Using a data target as the center of the circle, and using the distance of the data as the radius, can be used to calculate the information concentration value between data objects within adjacent jobs. The target object *c*_*a*_ is taken as an example to introduce and explain the collected data. If the object *c*_*b*_ is within its range, the similarity between *c*_*a*_ and *c*_*b*_ can be expressed as *d*(*c*_*a*_, *c*_*b*_). For the data object *c*_*a*_, the pheromone concentration value of *c*_*b*_ can be calculated as follows:

(3) $$\begin{array}{c} T_{ab}=\frac{Pc_{b}}{d\left(c_{a},c_{b}\right)}. \end{array}$$

The *Pc*_*b*_ in the formula can first establish the simplified pheromone diffusion model as shown in Figure 1 and then obtain it according to formula (2). It indicates that the data object *c*_*a*_ receives the pheromone concentration value of *c*_*b*_ within its scope, and *d*(*c*_*a*_, *c*_*b*_) indicates the similarity between *c*_*a*_ and *c*_*b*_.

The data object *c*_*a*_ calculates the pheromone concentration value of all data objects within its scope as follows:

(4) $$\begin{array}{c} T_{a}=\sum_{h\in H}\frac{Pc_{h}}{d\left(c_{a},c_{h}\right)}. \end{array}$$

In the formula, *h* represents all data objects in the scope *H* of the data object *c*_*a*_.

*Pheromone Enhancement and Volatilization*. It is supposed the enhancement parameter of pheromone is *Z* (*Z* > 0), and the volatilization parameter of pheromone is *y* (0 < *Y* < 1). Pheromone will volatilize over time. The volatilization amount of pheromone per unit time is *Y* times the original pheromone concentration value, and *Y* is the unit volatilization amount. With the migration of mobile agents, the pheromone concentration value on the link can be increased. If the mobile agent migrates from node a to node *b*(*b* ∈ *N*_*a*_), that is, the mobile agent migrates on the link *L*_*ab*_, Δ*T*_*ab*_ is the unit increment *Z*. The change in pheromone concentration over time is as follows:

(5) $$\begin{array}{c} T_{ab}\left(t+1\right)=\left(1-Y\right)T_{ab}\left(t\right)+\Delta T_{ab},\\ \Delta T_{ab}=\left\{\begin{array}{c} Z,\text{if agent transfer from a to b},\\ 0,\text{if agent transfer use other links}. \end{array}\right. \end{array}$$

The automatic topology discovery algorithm of penetration VR network usually adopts the automatic topology discovery scheme based on a mobile agent. This method solves the shortcomings of active routing strategies and demand-based routing strategies. In this article, based on mobile agents, we select network management nodes, introduce resident mobile agents, and divide the network into several subnets according to specific rules, so that nodes can only be transferred within the corresponding subnets. The network management node also introduces a mobile agent, and the generated mobile agent can collect all the node's automatic topology information carried by the mobile agent. It is a process to manage information resources. The immersive VR network information resources are managed in a number of related and orderly links, which form an organic whole. Intelligent management is to analyze the information resources in the immersive VR network through the three links of resource accumulation, resource arrangement, and resource utilization listed above [5].

When performing immersive VR network management analysis, we describe the basic information of the big data mapped by the network virtualization in the automatic topology discovery algorithm environment and transmit the big data packets of the network element network virtualization mapped from the source node through the network relay node. We create multiple network virtualization mapping propagation budget analysis and complete the network virtualization mapping budget analysis plan. Before planning the network virtualization mapping propagation budget analysis, the network environment should be modeled so that network virtualization mapping can better reflect the network, where the automatic topology discovery algorithm (also known as the unit solution) is used to establish the relevant network environment model. In the algorithm, the environment located in the big data of the network virtualization mapping is divided into areas or volumes through the unit decomposition method to obtain 2D or 3D meshes in the identical shape to form a network. The other elements in the environment are abstractly explained in units to construct a network environment that is easy to understand with big data mapped by network virtualization.

Regardless of the correct budget analysis between points and points, whether the initial node of the big data of the network virtualization mapping is separated at the exit, one of the initial nodes of the network virtualization mapping can be regarded as a typical immersive type at the exit VR network management analysis or a big data network virtualization mapping analysis with a constant network virtualization mapping as the end point of the initial node where the exit is not the initial node. In the case of using an automatic topology discovery algorithm to solve the virtual mapping analysis of a typical immersive VR network, all budget analysis points are taken as individuals in the group to select the matching function. For immersive VR network management analysis and ST-immersive VR network management analysis, only the optimal access sequence of the propagation budget analysis points can be obtained based on the automatic topology discovery algorithm. It is not a budget analysis and fails to comply with the analysis plan for the volume screening budget based on virtual mapping of the mobile network. Hence, an accurate analysis of the budget based on global planning is required through the automatic topology discovery algorithm [6].

The resource accumulation link includes information collection and information storage. At this stage, the community management system fully collects information resources in the immersive VR network; the resource sorting link includes information organization, information analysis, and user demand analysis after sorting out the analysis results. In this process, the system sorts out and analyzes the collected information in order to make the next intelligent recommendation and guide the rationalization of user behavior; resource utilization links include system recommendation, etc., use the analysis results to classify and filter the information that users may need, and actively recommend the essence of information to the user.

As a research hotspot in the field of cloud computing, network virtual resources are mainly aimed at reducing network mapping resources. This article analyzes the stability and network virtualization mapping, uses automatic topology discovery algorithms for the parameter optimization of the immersive VR network, and ensures that optimal solutions can be quickly obtained through not only factors but also those fully integrated in the visual field. The resources of the immersive VR network are initialized based on the automatic topology discovery algorithm to improve the global optimization capacity of the proposed algorithm. Users who join a permeable VR network can usually adjust their participation behavior as affected by the conduct of other community users. Based on the characteristics of the abovementioned user behavior, the administrator of the permeable VR network uses incentives and other methods to reasonably standardize and configure permeable VR. The virtualization of the network improves user participation. This management method is aimed at the intelligent management of the penetration-type VR network information resources. Permeable VR network virtualization and intelligent management are the analysis of user resources such as user behavior data and viewing history, mining user needs, predicting user behavior trends, and reflecting on the trend through information reorganization and regeneration. Individualized services are offered to users on demand so that they can enjoy the ultimate experience with added value.

The network management node periodically sends messages to the member nodes of the subnet and waits for a response. If the member node does not respond within the set time, indicating that the node is no longer in the subnet, the mobile agent deletes the node, updates the automatic topology information of the subnet, and returns the new automatic topology information to the network management node of the subnet. The network management nodes also realize the purpose of periodically exchanging the automatic topology information of each subnet and updating the automatic topology of the entire network.

*Implementation of the Algorithm*. Because the automatic topology discovery algorithm will have different types of network protocols and communication devices in the actual use process, but the data information calculation methods corresponding to different types of devices are different, in order to ensure that this communication device can be implemented under the top-level algorithm management and control, this article adopts a hierarchical structure mode in the automatic topology discovery algorithm cited in this article. The constructed hierarchical structure model is shown in Figure 2.

The communication equipment IP adopts a layer as the basis of the algorithm used in this article. In the layer, the IP address in the subnet is retrieved by using this function, and the corresponding subnet can be directly accessed via the subnet gateway IP. At present, there are many ways to retrieve the IP of subnet communication devices, such as the application of the Resolution Protocol contract. Here, the ICMP protocol is used to implement the echo response, or the ARP (Address Resolution Protocol) is used in the subnet. Through comparative analysis, this article selects the ICMP communication protocol as the data information of the echo response, because the data information echoed by the ICMP protocol used excludes the IP address other than the destination host to detect the existence of the IP address. In order to effectively solve this problem, this article can add an IP address by echoing the response data information, as shown in Figure 3. While the experimental data are transmitted through IP address, it is necessary to test the additional address to ensure that it is legit and that the IP field in the response message remains unchanged. The truthfulness of communication equipment can be ascertained from the IP address in this field.

In this case, the system problem can be displayed for the ICMP transmitted by the subnet at the same time, and the reply message can be obtained in the case of time-out according to another thread. The subnet protocol router that is directly connected to the network can be completed in a way that adapts to the addition of maintenance [7, 8].

*MAC Address Supplement Layer*. The main function of this layer is to correspond to the MAC address of the device in the subnet. In order to use the address translation data table, the connection between the main switch, switch, and router is required, and the MAC is mainly used. The main methods of extracting MAC addresses are ARP protocol and SNMP protocol.

*Discrimination Layer in communication equipment*. The same applies to routers, switches, and hosts using the algorithm of this article's automatic topology. The communication equipment type identification method used in this article is to identify and judge the equipment of this layer based on the data information of MIB-II sysServices. The sysServices data reflect the content of communication serves available in the protocol layer. For example, serves in the physical and data access layers are available through a two-layer switch. However, the sysServices has an identical value to the three-layer switch. Thus, the relevant sysService data should be provided to more effectively identify the two types of communication equipment.

We use an automatic topology algorithm to connect the analysis layer. This analysis layer can extract the data information of the communication equipment, complete the automatic acquisition, and then design a reasonable network topology. Automatic topology display layer: this layer allows the information obtained on the automatic topology data to be displayed in a graphical way. The algorithm flowchart is shown in Figure 4.

### 2.2. Immersive VR Network Management Analysis Process

*Immersive VR Network Request Mapping Scheme*. In order to maximize the life cycle of the network and reduce the poor packet loss and time delay in the transmission process of network data information, it is necessary to optimize the structure and topology of the multimedia network. This paper is based on the multimedia network real-time monitoring platform and proposes a multimedia network real-time monitoring method, according to the threshold of the multimedia network transmission node for early warning control; all multimedia network learning monitoring links need to be balanced; and the multimedia network real-time monitoring platform is used for multimedia network transmission delay control, which can effectively enhance the data real-time monitoring capability. We reduce the packet loss rate of data transmission and improve transmission performance. In the routine application, the imbalance, turbidity, and instability of network virtualization mapping are essential. Optimization of the support-vector regression model can be performed based on the chaotic particle swarm and artificial fish swarm optimization algorithms. Three different groups of time particle data are selected from the MAWI dataset to establish the analysis model for network mapping combined with examples and detailed analysis. Nodes and link elements have a certain impact on immersive VR network management analysis. In order to simplify the mapping analysis process and accurately describe it, network nodes generally need to fully consider various link information such as CPU, memory, and location information.  Figure 5 shows the mapping scheme of the underlying network using the immersive VR network.  Figure 5(b) is the lower part of the network link. The numbers represent the bandwidth information that can be used by the link, and the numbers in the rectangle around the node represent the CPU and memory resource utilization that can be used [9, 10].

In the network environment, we use the automatic topology discovery algorithm to analyze the network virtualization map propagation budget. In the process of promoting the plan, the OPEN/CLOSE tables are constructed, in which the OPEN table is attached to the initial node upon initialization, and the CLOSE table is void, with the initial node as follows:

(6) $$\begin{array}{c} f\left(s\right)=h\left(s\right), \end{array}$$

where *f* (*s*) is the initial assessment function; *h* (*s*) denotes the estimated interval between the initial and end nodes.

If the OPEN list is void without a target location, the search is suspended without valid budget analysis; otherwise, the following steps are repeated until the target node is secured:

(1) In the OPEN table, the node with a smaller value (*f*) is selected and added to the CLOSE table, and the corresponding value is deleted from the OPEN table. If the node (*q*) has the minimum value (*f*) in the neighboring nodes at the initial node, this initial node is deemed as the parent node.
(2) All the neighboring nodes of *p* are calculated. If the neighboring node *u*_*i*_ is used for explanation, *f*(*u*_*i*_), *h*(*u*_*i*_), and *g*(*u*_*i*_) are identified. Here, *g*(*u*_*i*_) is used to describe the interval between the selected and target nodes, which can be determined as follows.
  ① For terminal station *u*_*i*_, we exit 3D technology algorithm for reconstruction. Starting with the terminal, we trace back to the initial node from the parent to analyze the budget for batch picking of network virtualization mapping.
  ② For inaccessible point *u*_*i*_, we skip and proceed to the next step.
  ③ For *u*_*i*_ in the CLOSE table, we skip and proceed to the next step.
  ④ For non-OPEN/CLOSE table point *u*_*i*_, we add it to the OPEN table as a parent node.
  ⑤ For *u*_*i*_ in the OPEN table, we obtain the value for *g* by analyzing the new budget. If it is minimum, *p* is considered a parent node of *u*_*i*_, while upgrading *f*, *h*, and *g*; otherwise, it remains unchanged.

We save the search path and trace from the parent to the initial node.

*Internet Control Message Protocol (ICMP)*. There are reports in the ICMP protocol used that errors or exceptions have occurred in the host or the router used, but the ICMP protocol is not an upper-layer protocol, but is mainly a type of IP layer protocol. ICMP messages can be used for data messages at the network layer and together with the beginning of the data message constitute the transmission of IP data messages [11]. ICMP has different types of messages, which can be roughly divided into ICMP error messages and ICMP query messages. The two messages used in the message algorithm are mainly response requests and responses, and the corresponding message format is shown in Figure 6. The response request/response is mainly to test the feasibility and connectivity of the sink. Request is to send a response request to a specific sink, and the response sent by the sink includes a copy of any data area requested, as shown in Figure 6.

The response request and response are all transmitted in the network according to the expression form of the IP data message. If the data of the response data copy dataset and the request process can be smoothly obtained, it can not only indicate that the sink machine can reach it but also further explain the data. The message has a normal function in the transmission system.

*SNMP (Simple Network Management Protocol)*. The SNMP is mainly to ensure that the network management station NMS can implement detection and network element management and control in a simple and effective mode. Its basic structure is mainly divided into the following three parts:

1. The service request information of the application software tool entity that the management station can receive forms the SNMP data message and sends the data information to the agent in real time.
2. The management data information database stores management parameters under different types of targets. The structure of the management information database is mainly defined by SMI, and the corresponding data information structure is similar to an inverted tree. Among them, each variable in the management data information database is also identified by all nodes that pass from the root of the tree to the variable.
3. The agent stays in the management and control of different types of data, maintains and updates the local agent data information, processes the MIB variable acquisition request message sent from the management station, and wants to send the data message from the management station after the identity check. This corresponding message mainly contains the variables requested by the management station or the corresponding error data information.

The SNMP protocol switches the data information between the management station and the agent and the agent port 161, while the port of the management station is 162, SNMP Western medicine adopts the polling mode, and the report of the trap mechanism also illustrates special emergency situations, so SNMP can be used as a network management protocol with high practical value. In addition, because the SNMP protocol is a wireless connection based on UDP, you can use the SNMP protocol to obtain unstable types of nonconnection services. If you want to obtain better network quality, the network management process needs to be placed at a higher level. We perform the connection operation.

The SNMP protocol is mainly implemented for five protocol units, but under this algorithm, there are only some types of messages such as Get-Request, Get-Next-Request, and Get-Response.

Immersive VR network management system structure is a working group of immersive VR network management by IETF. In this paper, network services are described and measured by a general framework [12], and immersive VR network management is proposed to control the risks in real time according to the framework using the monitoring platform of the immersive VR network.  Figure 7 shows the management system architecture of the immersive VR network. The monitoring system includes 4 subsystems: input of modular rules, collection of flows, data analysis, and database.

In this management system, the rule set in the input system is used for business collection, and filters and aggregates the business of the network with thousands of real-time network services. The effective data obtained are stored in the database and forwarded for data analysis. The valid data are processed by the data analysis system, and changes in network services are predicted to adjust distribution information and manage network actions.  Figure 8 shows the flow of the system management system.

The packets intercepted in the shared media network cannot be timely processed because any packet transmitted via the network is larger than that required by the network segment service in the hardware configuration. Where the network segment is equipped with the server for traffic analysis and externally interconnected and the equipment NIC in the “hybrid” mode, it is possible to capture any packet of IP data accessing the network. With the required information such as source and destination address, data volume, and application protocol, analysis and consolidation can be performed on IP packets. This method is superior in that no change in the structure of the network, increase in network load, or occupation of network resources is required [13], nor does it extend the network lag or influence the usage experience of users.

The proposed sniffer method by raw socket is simple, where only the packets containing no frame data on the IP layer are deleted without the necessity to comply with special requirements. The network traffic management system is analyzed, and it can be seen that the overall network traffic is mainly in the penetration VR network monitoring platform in real time, where any traffic adjustment basically reflects the overall change of the network traffic in the penetration VR network. The real-time monitoring platform traffic can replace the total traffic to analyze network performance. That is, raw socket can be used to obtain traffic information [14]. As shown in Figure 9, the initialization network in the monitoring node link monitoring system is used to establish the set of cluster head vectors at the node of multimedia sensing data under the multimedia. The dataset is further divided into several 2D subareas (Ak) by time window width, where Ak represents a 2D information entropy group compliant with *A*1, *A*2, Ak = *A*. *D*_*n*_|*d*_*n*−max_ − *d*_*n*−min_| · (1/*K*)…. Figure 9 shows the layout for channel allocation of two relay nodes monitored by multimedia.

Where the SN and the sink of the immersive VR network have a certain space, initialization is performed for *k* = 1. The distribution set at the sensor node monitored by multimedia is *S* = {*s*_1_, *s*_2_,…, *s*_*n*_}, and the uniform layout method is used to establish the double-layer relay node. The configuration equation for feature distribution can be obtained as follows:

(7) $$\begin{array}{c} f\left(v_{i},v_{j}\right)\geq 0,\\ \sum f\left(v_{0},v_{k}\right)=0\left(1\leq k\leq n+m\right),\\ \sum f\left(v_{i},v_{k}\right)=0\left(1\leq k\leq n\right)\\ \sum \left(f\left(v_{i},v_{k}\right)-f\left(v_{h},v_{j}\right)\right),=0,\left(n+1\leq k\leq n+m,1\leq h\leq n+m\right). \end{array}$$

The 2D entropy feature data corresponding to the sensor node in the cluster are extracted according to the specific configuration design at the corresponding immersive VR network node in the following steps, which can reduce the computational overhead of the multimedia [15].

Step 1: In the immersive VR network, geographic coordinates of SN and sink are input to start immersive VR network monitoring.
Step 2: The sleep time is confirmed. SN and sink distance *d* = {*d*_1_, *d*_2_,…, *d*_*n*_} in the information center are sorted, with the set *S* = {*s*_1_, *s*_2_,…, *s*_*n*_} corresponding to the location distribution of multimedia sensor node cluster in the monitoring area.
Step 3: *k* = 1 is initialized to identify the pseudo-random adaptive sequencing of multimedia sensors at the current position, where Tag = 1.
Step 4: If *d*_*k*_ ≥ *d*_0_ is satisfied, then Tag (*k*) = 1, the data information cluster fusion center can be obtained to the optimal position and, at the same time, proceed to step 5; otherwise, the algorithm is terminated.
Step 5: The maximum hop for the learning factor sk.count_max(*s*, *v*)*χ*_*k*_ in the immersive VR network is associated with the sensing network route itself and Tag (*k*) = 0.
  (8) $$\begin{array}{c} \left|\frac{d\left(s_{k},v_{0}\right)}{d_{0}}-\chi_{k}\right|\leq 0.5. \end{array}$$

## 3. Application and Testing

In the test experiment of this article, the selected programming language is VC++2005 software; using an object-oriented design method, the proposed automatic topology algorithm is modularized on this platform; and at the same time, it is applied to the integrated network management platform for testing. The network management platform of the experiment process is based on the automatic topology algorithm selected in this article, and realizes real-time monitoring of the entire network communication equipment to ensure that the network can be stably and normally used. Test results in different types of network environments and communication equipment show that the use of automatic topology discovery algorithms can accurately and quickly design the network structure, and at the same time can run better. As indicated in Figure 10, among them, the gateway router of the subnet 192.168.1.^*∗*^ subnet 192.168.2^*∗*^ is generally connected by the internal switch of the subnet, but the gateway router of the subnet 192.168.2^*∗*^ subnet 192.168.3^*∗*^ adopts the direct connection method.

In order to test the real-time management performance of the immersive VR network proposed in this paper, the simulation software MATLAB is used to realize the test path plan and target positioning model of the immersive VR network topology, the network management coverage is set to 2000 × 2000, the topological number is 200, the sink topological number is 10, the source topological number is 25, and the multimedia data information transmission wave rate is set to 1 Mboud. The information collection sampling speed is 12 ms/s, and this method is used for immersive VR network monitoring, as shown in Figure 11, and the sample sequence output from the monitoring topology.

The sequence samples shown in Figure 8 are set as the SINR threshold of the test subject. *β* = intensity of background interference data. Multimedia information fusion and 2D entropy feature extraction are performed using the sensor topology fusion tracking scheme in the cluster. Figure 11 shows the information fusion result.

Analyzing Figure 12, we can see that the immersive VR network learning is carried out by the method of this manual, the fusion effect of multimedia sensing information is better, and the output multimedia information has a higher interference prevention ability. The maximum entropy matching degree value of the test monitor is based on the set threshold matching degree value Hgt = 3. As shown in Figure 12, it is shown that the monitoring link of the immersive VR network manager equalizes the calculation result of the maximum entropy matching value.

The maximum entropy is 3.2982. The immersive VR network management designed in this paper has link balance to ensure the accuracy and real time of information management. Finally, different methods are tested to measure the loss rate of network management, and the comparison result is shown in Figure 13.

## 4. Discussion

The proposed distributed network management system adopts the structure of several subcontrol centers under the general control center, further divides the responsibilities and rights of the backbone network and the park network, and realizes data distribution and management distribution according to the principle of data and basic management nearby. The distributed network management system has fully considered the efficiency, scalability, flexibility, security, and visibility of the user interface. At present, this paper still has some problems to be solved. For example, the construction of the subcontrol center is rather complicated, the topology exploration also adopts the physical topology that can realize deep measurement and full meaning, and the design and implementation of many algorithms and strategies in traffic analysis are still to be solved. These are all the problems that need to be solved in the next step. After all, we have taken the first step to make a pleasant progress. In the future, we will continue to explore the implementation strategy of more efficient and effective implementation, the Xin II algorithm, and constantly improve the function and performance of the network management system.

## 5. Conclusions

For the purpose of optimizing the network and physical layer topology in the switched internet, an automatic topology discovery algorithm for immersive VR network management analysis is proposed in this paper, where the entire network is divided into multiple independent networks. The modules in each module realize the effective management of the network. The results of the experiment indicate that the proposed method can effectively address the issue of the traditional method in dealing with the automatic topological structure separation between the network layer and the physical layer, and the management is invalid, which improves the efficiency of network management analysis.

## Figures and Tables

**Figure 1:** Simplified pheromone diffusion model.

**Figure 2:** Block diagram of the hierarchical structure model.

**Figure 3:** ICMP echo response message format diagram.

**Figure 4:** Algorithm flowchart.

**Figure 5:** The mapping scheme of immersive VR network requests. (a) Virtual network request. (b) Underlying network.

**Figure 6:** Response request/response (type 0) message format.

**Figure 7:** Immersive VR network management system structure.

**Figure 8:** System process.

**Figure 9:** Channel allocation layout at two-layer relay nodes monitored by multimedia.

**Figure 10:** Automatic topology discovery diagram of a company's network.

**Figure 11:** Sample sequence output from immersive VR network management topology.

**Figure 12:** Multimedia sensor information fusion results.

**Figure 13:** Calculation results of the maximum entropy fitness value.

## Data Availability

The data used to support the findings of this study are available from the corresponding author upon request.
